# Influence of organic manures on soil nutrient content, microbial population, yield and quality parameters of pomegranate (*Punica granatum* L.) cv. Bhagwa

**DOI:** 10.1371/journal.pone.0266675

**Published:** 2022-04-18

**Authors:** Ramesh Chand Choudhary, H. L. Bairwa, Uttam Kumar, Talha Javed, Muhammad Asad, Kanhaiya Lal, L. N. Mahawer, S. K. Sharma, Pushpendra Singh, Mohamed M. Hassan, Ali A. Abo-Shosha, Rajinikanth Rajagopal, Nader R. Abdelsalam

**Affiliations:** 1 Department of Horticulture, Rajasthan College of Agriculture, Maharana Pratap Agriculture University and Technology, Udaipur, Rajasthan, India; 2 College of Plant Protection, Fujian Agriculture and Forestry University, Fuzhou, China; 3 College of Agriculture, Fujian Agriculture and Forestry University, Fuzhou, China; 4 College of Life Science, Fujian Agriculture and Forestry University, Fuzhou, China; 5 Department of Agronomy, Dr. Rajendra Prasad Central Agricultural University, Pusa, Samastipur, Bihar; 6 Department of Biology, College of Science, Taif University, Taif, Saudi Arabia; 7 Genetics Department, Faculty of Agriculture, Kafrelsheikh University, Kafr El-Sheikh, Egypt; 8 Sherbrooke Research and Development Center, Agriculture and Agri-Food Canada, QC, Canada; 9 Agricultural Botany Department, Faculty of Agriculture (Saba Basha), Alexandria University, Alexandria, Egypt; Kyonggi University, REPUBLIC OF KOREA

## Abstract

During the last era in India, the use of chemical fertilizer has increased tremendously. The excessive use of these chemicals leads to the degradation of soil quality, health, as well as nutritional status. These are also causing a degradation of human health. This experiment was conducted during *Mrig Bahar* (July to December) during two consecutive years (2019–2020)in a randomized block design with three replications in which six-year-old 42 pomegranate plants were tested with 14 treatments of different organic manures. Findings showed that in the various treatments, the organic combination T_13_-Jeevamrut 16.08 L plant^-1^ + Vermicompost 24.79 kg plant^-1^ had a significant effect on the nutritional status (available nitrogen, available phosphorus, and available potassium) and microbial population (fungi, bacterial, and actinomycetes count). In addition, T_13_-*Jeevamrut* 16.08 L plant^-1^ + Vermicompost 24.79 kg plant^-1^ found a significant effect on fruit yield characteristics like fruit plant^-1^ (122.00), fruit yield (17.38 kg plant^-1^), fruit weight (192.50 g) and fruit quality characteristics such as fruit juice percent (52.92%), and total sugar (11.92%).

## Introduction

After the start of green-evolution in India, farmers used chemical fertilizers to increase the production and productivity of different crops. The excessive use of chemical fertilizers has negatively impacted the soil fertility, biodiversity, quality of the produce and human health. In addition, it also increased soil acidity, deteriorated soil physical condition, decreased organic matterand created micronutrient deficiencies. To solve these problems, the future of agriculture should be diverted to organic farming. Because organic manure not only provides vital nutrients (including micronutrients), but it also improves the physical and biological state of soils, improves aeration, and provides improved root growth and production opportunities. It is a recommended practice for low-chemical-input sustainable gardening. Increased nutritional availability [1], soil physical conditions and enzymatic activity have been reported by vermicompost application in fruit crops. Vermicompost is high in organic carbon, which is important for soil fertility, and it includes all of the required plant nutrients in the right amounts [2]. As a result, it is a well-balanced plant food. It also contains biological compounds that aid in the growth of plants and the prevention of plant diseases [3]. The use of vermicompost improves the soil’s ability to hold water while also increasing the rate of water intake into the soil. It improves the colour, smell, taste, and flavour of fruits as well as their shelf life. Organic manure help to maintain and improve soil quality and productivity at a low cost of input. Organic nutrient sources help to preserve soil health by keeping a balance of organic matter and soil microflora, which results in improving the soil’s physical, chemical, and biological qualities [4]. The use of vermicompost in conjunction with mineral fertilizers has yielded promising results in terms of crop productivity and soil health [5]. The use of green manures such as vermicompost, FYM, and sun hemp (Crotolaria juncea L.) in combination with chemical fertilizers has resulted in the preservation of soil’s physical, chemical, and biological qualities [6]. In addition to enhanced microbial establishment, FYM enables the formation of extra humus content [7].

In soils with structural problems or nutrient deficits, compost improves drainage and moisture absorption. They also allow farmers to boost crop output, improve plant growth by adding critical nutrients, deploy in a variety of soil types, reduce runoff, and reap financial rewards. Organic composts have been demonstrated to boost the flowering and growth of freshly planted trees, as well as fruit production, in apple orchard soils [8]. According to Boraiah *et al*. (2017) [9], Jeevamrut enhances biological activity in the soil and increases the availability of nutrients to the crop. Greater microbial load and growth regulators may have increased soil biomass, allowing for the accessibility and absorption of applied and native soil nutrients, resulting in improved crop growth and production.

Pomegranate (*Punica granatum* L.) cv. Bhagwa is a widely produced horticultural crop in Rajasthan, India’s south-west. With increasing demand, pomegranates with a great market value can produce nutrient-rich fruits that have enormous benefits for humans. This fruit crop can withstand drought, salinity, and a harsh winter, as well as thrive in rainfed conditions. Because of the tremendous commercial worth of this fruit, its cultivation is gradually rising. Consumer interest in its eating stems in part from the organoleptic qualities of the arils (seeds) as well as the health benefits [10]. As a result, the current study aimed to evaluate the effects of 14 different organic manure treatments with the following goals: (ii) investigate the impacts of multiple organic manures on important soil nutrients and the microbial population of the soil; (ii) distinguish the impact of different organic manures on pomegranate yield and quality parameters; and (iii) frame out the best organic manure to optimize pomegranate yield and quality. Based on our aims, we hypothesized that that different organic manures would affect soil chemical properties, microbial populations, and pomegranate yield responses differently. The research will provide quantitative insight into pomegranate cultivation management for growth and productivity.

## Material and methods

### Description of study site

The experiment was carried out at Technology Park, CTAE and laboratories of the Department of Horticulture, Rajasthan College of Agriculture, MPUAT, Udaipur (Rajasthan) located at 582.17 m above mean sea level with coordinates of 24° 34´ N latitude and 73° 42´ E longitude. The experimental site’s soil has pH 8.5, with clay loam texture, medium organic carbon (OC) (0.644%), and is low in available nitrogen (AN) (272.68 kg ha^-1^), available phosphorus (AP) (23.90 kg ha^-1^) and available potassium (AK) (292.82 kg ha^-1^). The weekly meteorological parameters of the experimental site were recorded during the crop seasons of 2019 and 2020. The maximum temperature (42.90 & 40.80°C) and relative humidity (94.3 & 95.7%) were recorded in 2019 and 2020, respectively. The minimum temperature (4.7 & 3.8°C), relative humidity (11.3 and 19.9 mm) and annual rainfall (1160.6 and 862.7 mm) were recorded during 2019 and 2020, respectively. They are presented in Fig 1.

**Fig 1:** Mean weekly weather parameters during cropping seasons in both the years.

### Trial design

A field experiment has been conducted for two consecutive years between 2019 and 2020 to investigate the effect of adding different types of organic manure amendments on the nutritional content and microbial population of a crop. The Randomized Block Design was used for the layout of experiments. There were 14 treatment combinations [T_1_-Control, T_2_- Recommended Dose of Fertilizer (RDF) (600: 200: 200g NPK/Plant/year) the source of NPK was urea, DAP and MAP respectively, T_3_- Farm Yard Manure (FYM) (120.72 kg/plant), T_4_- Compost (54.10 kg/plant), T_5_- Vermicompost (49.58 kg/plant), T_6_- Narayan Deotao Pandharipande (NADEP) Compost (70.83 kg/plant), T_7_- Jeevamrut (32.17 L/plant), T_8_- FYM (60.36 kg/plant) + Compost (27.05 kg/plant), T_9_- FYM (60.36 kg/plant) + Vermicompost (24.79 kg/plant), T_10_- FYM (60.36 kg/plant) + NADEP compost (35.41 kg/plant), T_11_- Jeevamrut (16.08 L/plant) + FYM (60.36 kg/plant), T_12_- Jeevamrut (16.08 L/plant) + Compost (27.05 kg/plant), T_13_- Jeevamrut (16.08 L/plant) + Vermicompost (24.79 kg/plant) and T_14_- Jeevamrut (16.08 L/plant) + NADEP (35.41 kg/plant)] with 3 replications and in each replication one tree served as a treatment unit. Thus 42 trees were selected for the experiment.

### Soil sampling and analysis

Soil samples with the help of bucket auger were taken from all selected plants at a depth of 0–90 cm. These samples were air dried before being crushed with a wooden pestle and mortar and sieved at a size of 2 mm. The following tests were performed on these samples. Alkaline permanganate method for chemical examination of soil, such as available nitrogen [11], available phosphorus with Olsen’s method [12] and available potassium was estimated through flame-photometer [13]. Organic carbon content was determined by rapid titration method [14]. Microbial population was detected by using serial dilution plate method [15]. A reconnaissance of the experimental field was conducted, and the soil samples were taken. After preparing the soil samples for microbial population, the soil (30–60 cm depth) was collected in a polythene bag and stored at 40°C. On yeast extract mannitol agar, the initial microbial population was quantified using the serial dilution pour plate technique (YEMA).

### Yield and quality characteristics

#### Fruit plant^-1^ (Number)

Each plant’s total number of fruits harvested were counted.

#### Fruit yield (kg plant^-1^)

Each plant’s fruits were weighed with a weighing balance, and the yield per treatment and replication was calculated.

#### Fruit weight (g)

Five marketable fruits were selected from each treatment and replication, and their fresh weight was measured to determine the average fruit weight.

#### Fruit cracking percent

Count the cracked fruits and divided by total number of fruits and then multiplied by 100.

#### Rind thickness (mm)

Rind thickness was measured with the help of vernier calipers. Average of five fruits per treatment was taken to record the rind thickness.

#### Juice percent (%)

100 g fleshy aril was taken and juice was extracted using juicer and the weight of juice was measured in each treatment separately.

#### Acidity (%)

A fruit sample of five grams was macerated in a pastel mortar with distilled water and the volume was made up to 10 ml. The extract was then filtered through a rough filter paper and an aliquot of 2 ml was taken for titration against the N/10 NaOH solution using two drops of 1.0 percent phenolphthalein solution as an indicator. The endpoint of titration appeared as a light pink color. The acidity was calculated using the following formula based on the NaOH used, and the results were expressed as gram citric acid per 100 g of sample [16].


$$Acidity\;percent=\frac{Titre\;x\;acid\;factor\;x\;100}{10\;ml\;juice}$$

#### Total sugar (%)

In a test tube, 5 ml of diluted juice extract and 4 mL of concentrated HCl were added to it. Then they covered them with aluminum foil and kept them for 15 minutes at 68°C in a boiling water bath. After cooling the test tubes under tap water, the acidity was neutralized by adding anhydrous sodium carbonate till the effervescence stopped. The final volume was set at 50 ml with distilled water and Using starch as an indicator, the liberated iodine was titrated with a 0.01N sodium thiosulphate solution. The disappearance of the blue colour and the appearance of a milky white colour was the end point. A blank was also run simultaneously. The results were calculated using the following formula and expressed in percent.

% Total Sugars = Fehling’s solution factor ×100×Dilution The volume of sample used ×1000

#### Statistical analysis

The data were analyzed statistically using Prism-8.0.1, using one-way ANOVA per time and multiple comparison tests (LSD and Dunnett’s T3) to find significant differences (0.05). For visualization and tables, we utilized Prism-8.0.1, and Microsoft Excel-2016, respectively.

## Results

### Nutritional content of soil

Different organic manure treatments had a significant effect on the available NPK status of soil, as shown in Table 1 and Fig 2, along with these organic carbon (%) was also found to be significant. The data showed that the application of organic combination level T_13_-Jeevamrut 16.08 L plant^-1^ + Vermicompost 24.79 kg plant^-1^ has recorded maximum AN (290.07 kg ha^-1^), AP (25.58 kg ha^-1^) and AK (315.58 kg ha^-1^) content in soil as comparison to the control (T_1_). Compared to T_1_, soil OC content greatly increased under T_13_ and T_2_ treatmentsin different phases (Fig 1D). Similarly, for AP and AK, T_13_ treatment followed by T_2_showed significant (P < 0.05) effects over control (Fig 2B and 2C). Soil AN and AK contents were greater in year 2020 under maximum of treatments (Table 1, Fig 2A–2C). For soil AN, overall significant trend in both years was as follows: T_13_> T_12_> T_11_> T_10_> T_2_> T_3_. For soil AP, overall most significant trend in both years was as follows: T_13_> T_12_> T_2_. For soil AK, overall most significant trend in both years was as follows: T_13_> T_12_> T_8_> T_2_> T_3_. For soil OC, overall most significant trend in both years was as follows: T_13_> T_12_> T_9_> T_2_> T_3_.

**Fig 2:** The effect of different organic manure treatments on soil chemical properties, where (**a**) Available nitrogen (AN); (**b**) Available phosphorus (AP); (**c**) Available potassium (AK); d) Organic carbon (OC). Various asterisk on bars show the significant differences (*P* < 0.05) with vertical bars as standard errors (*n* = 4) (****>***>**>*>ns).

**Table 1:** Effect of organic manures on available nutritional content (kg ha^-1^) in soil.

Treatments	Available Nitrogen (kg ha^-1^)			Available Phosphorus (kg ha^-1^)			Available Potassium (kg ha^-1^)			Organic carbon (%)		
	2019	2020	Pooled	2019	2020	Pooled	2019	2020	Pooled	2019	2020	Pooled
T_1_	271.39	270.42	270.90	23.50	23.12	23.31	292.02	291.67	291.85	0.641	0.639	0.640
T_2_	279.24	285.81	282.52	24.96	25.78	25.37	310.45	312.20	311.33	0.642	0.642	0.642
T_3_	275.12	277.98	276.55	24.33	25.00	24.66	302.14	303.07	302.60	0.648	0.649	0.648
T_4_	275.32	279.45	277.39	24.50	25.25	24.88	305.92	307.22	306.57	0.643	0.643	0.643
T_5_	276.82	280.14	278.48	24.75	25.50	25.13	308.11	309.34	308.73	0.650	0.651	0.651
T_6_	267.57	274.11	270.84	23.50	24.00	23.75	294.68	296.34	295.51	0.644	0.645	0.645
T_7_	269.28	276.41	272.84	23.67	24.33	24.00	295.33	297.20	296.27	0.648	0.649	0.649
T_8_	276.82	282.47	279.65	24.83	25.67	25.25	308.79	310.11	309.45	0.647	0.647	0.647
T_9_	277.57	283.65	280.61	24.90	25.75	25.33	310.09	312.13	311.11	0.650	0.652	0.651
T_10_	274.82	276.44	275.63	24.00	24.75	24.38	297.84	299.12	298.48	0.647	0.648	0.648
T_11_	280.57	289.14	284.86	25.00	25.85	25.43	311.12	312.87	312.00	0.643	0.643	0.643
T_12_	282.82	291.66	287.24	25.06	25.90	25.48	312.96	314.14	313.55	0.644	0.647	0.646
T_13_	285.48	294.66	290.07	25.15	26.01	25.58	314.27	316.89	315.58	0.647	0.649	0.648
T_14_	274.32	275.36	274.84	23.90	24.50	24.20	298.45	300.87	299.66	0.641	0.643	0.642
**SEm±**	**3.27**	**4.23**	**2.47**	**0.42**	**0.43**	**0.28**	**4.28**	**4.27**	**2.80**	**0.01**	**0.01**	**0.01**
**CD (P = 0.05)**	**9.52**	**12.28**	**7.02**	**1.22**	**1.25**	**0.79**	**12.45**	**12.40**	**7.94**	**NS**	**NS**	**NS**

Initial value of available Nitrogen = **272.68,** Phosphorus = **23.90 kg ha**^**-1**^, Potassium = **292.82 kg ha**^**-1**^ and Organic carbon = **0.644%.**

### Microbial population of soil

It is found that the different organic manure treatments had a significant effect on soil microbial properties, which are fungi, bacteria, and actinomycetes, during the both the years (Table 2 and Fig 3). The pooled data showed maximum availability of fungi count (23.68 x10^4^ CFU/g), bacterial count (62.68 x10^6^ CFU/g) and actinomycetes count (27.77 x10^4^ CFU/g) were observed with treatment organic combination level T_13_-Jeevamrut 16.08 L plant^-1^ + Vermicompost 24.79 kg plant^-1^ as compared to T_1_-control (minimum) and T_2_-RDF (600: 200: 200 g NPK plant^-1^). For Fungi, overall significant trend in both years was as follows: T_13_> T_12_> T_11_> T_8_> T_2_> T_9_. For Bacteria, overall most significant trend in both years was as follows: T_13_> T_12_> T_11_> T_9_> T_2_> T_4_. For Actinomycetes, overall most significant trend in both years was as follows: T_13_> T_12_> T_11_> T_9_> T_2_>T_4_> T_3_> T_5_.

**Fig 3:** The effect of different organic manure treatments on soil microbial populations, where (**a**) Fungi; (**b**) Bacteria; (**c**) Actionmycetes. Various asterisk on bars show the significant differences (*P* < 0.05) with vertical bars as standard errors (*n* = 4) (****>***>**>*>ns).

**Table 2:** Effect of organic manures on fungi, bacteria and actinomycetes population in per gram of soil.

Treatments	Fungi (x10^4^ CFU/g)			Bacteria (x10^6^ CFU/g)			Actinomycetes (x10^4^ CFU/g)		
	2019	2020	Pooled	2019	2020	Pooled	2019	2020	Pooled
T_1_	21.36	21.50	21.43	57.98	58.00	57.99	25.56	25.67	25.62
T_2_	22.85	23.33	23.09	60.36	61.00	60.68	26.75	27.33	27.04
T_3_	22.75	23.05	22.90	59.36	60.20	59.78	26.50	27.00	26.75
T_4_	22.80	23.20	23.00	60.17	60.67	60.42	26.65	27.12	26.89
T_5_	23.00	23.67	23.34	60.72	61.33	61.02	26.90	27.50	27.20
T_6_	21.67	21.90	21.79	58.05	58.33	58.19	25.67	25.75	25.71
T_7_	22.00	22.25	22.13	58.30	58.67	58.49	25.75	26.12	25.94
T_8_	23.04	23.80	23.42	61.37	62.00	61.68	27.00	27.67	27.34
T_9_	23.10	23.85	23.48	61.87	62.33	62.10	27.15	27.85	27.50
T_10_	22.50	22.84	22.67	58.61	59.33	58.97	26.33	26.85	26.59
T_11_	23.17	23.96	23.57	62.12	62.50	62.31	27.25	27.97	27.61
T_12_	23.21	24.00	23.61	62.25	62.67	62.46	27.30	28.04	27.67
T_13_	23.29	24.06	23.68	62.36	63.00	62.68	27.42	28.12	27.77
T_14_	22.33	22.60	22.46	58.56	59.00	58.78	26.00	26.50	26.25
**SEm±**	**0.39**	**0.39**	**0.26**	**0.80**	**1.02**	**0.60**	**0.41**	**0.46**	**0.29**
**CD (P = 0.05)**	**1.12**	**1.15**	**0.73**	**2.34**	**2.97**	**1.71**	**1.18**	**1.34**	**0.81**

Initial value of Fungi = **20.88 x10**^**4**^ **CFU/g**, Bacteria = **56.68x10**^**6**^ **CFU/g** and Actinomycetes = **25.47x10**^**4**^ **CFU/g.**

### Yield characteristics

The ultimate goal of pomegranate producers is to achieve maximum profits per unit area per unit time. With the use of organic manures and inorganic fertilizer, the crop’s fruit output attributes improved dramatically (Table 3 and Fig 4). The application of treatment T_2—_recommended dose of fertilizer (RDF-600: 200: 200 g NPK plant^-1^) has recorded the maximum number of fruits (121.33, 125.00 and 123.17) plant^-1^; fruit yield (17.18, 18.01 and 17.59 kg plant^-1^); and fruit weight (189.70, 199.65 and 194.68 g), which was statistically at par with organic treatment combination T_13_—*Jeevamrut* 16.08 L plant^-1^ + Vermicompost 24.79 kg plant^-1^; fruit yield (17.02, 17.74 and 17.38 kg plant^-1^); and fruit weight (188.03, 196.97 and 192.50 g) during both the experimental years. For both fruit yield and fruits per plant, overall significant trend in both years was as follows: T_2_> T_13_> T_12_> T_11_> T_8_> T_9_. For fruit weight, overall most significant trend in both years was as follows: T_2_>T_13_> T_12_> T_11_> T_9_ > T_8_. For rind thickness, overall most significant trend in both years was as follows: T_2_>T_13_> T_12_> T_11_> T_9_ > T_8_.

**Fig 4:** The effect of different organic manure treatments on soil chemical properties, where (**a**) Fruit yield; (**b**) Fruits per plant; (**c**) Fruit weight; d) Rind thickness. Various asterisk on bars show the significant differences (*P* < 0.05) with vertical bars as standard errors (*n* = 4) (****>***>**>*>ns).

**Table 3:** Effect of organic manures on fruit quality characteristics of pomegranate cv. ‘Bhagwa’.

Treatment	Fruits plant^-1^ (Number)			Fruit yield (kg plant^-1^)			Fruit weight (g)			Fruit cracking percent (%)		
	2019	2020	Pooled	2019	2020	Pooled	2019	2020	Pooled	2019	2020	Pooled
T_1_	101.00	102.00	101.50	14.91	15.35	15.13	150.58	157.70	154.34	3.93 (2.10)	2.90 (1.70)	3.42 (1.90)
T_2_	121.33	125.00	123.17	17.18	18.01	17.59	189.70	199.65	194.68	2.64 (1.77)	1.33 (1.18)	1.99 (1.48)
T_3_	106.00	109.67	107.83	15.50	16.00	15.75	160.22	169.33	164.77	0.63 (1.06)	2.80 (1.68)	1.71 (1.37)
T_4_	108.67	111.00	109.83	15.57	16.08	15.83	163.01	171.68	167.35	0.69 (1.09)	2.67 (1.65)	1.68 (1.37)
T_5_	110.33	114.00	112.17	15.90	16.65	16.28	171.32	181.46	176.39	1.11 (1.27)	0.00 (0.71)	0.55 (0.99)
T_6_	103.00	105.00	104.00	15.01	15.51	15.26	155.01	163.55	159.28	0.57 (1.03)	0.93 (1.15)	0.75 (1.09)
T_7_	104.00	107.00	105.50	15.17	15.63	15.40	156.42	165.21	160.82	0.59 (1.04)	3.18 (1.77)	1.89 (1.41)
T_8_	112.00	115.67	113.83	16.19	16.86	16.53	173.21	182.12	177.67	2.16 (1.63)	0.00 (0.71)	1.08 (1.17)
T_9_	114.00	117.00	115.50	16.40	17.10	16.75	176.52	185.69	181.11	2.20 (1.64)	0.00 (0.71)	1.10 (1.18)
T_10_	105.00	107.67	106.33	15.37	15.86	15.62	159.33	167.67	163.50	0.61 (1.05)	2.75 (1.67)	1.68 (1.36)
T_11_	116.00	119.00	117.50	16.75	17.25	17.00	181.76	190.54	186.15	2.30 (1.67)	0.00 (0.71)	1.15 (1.19)
T_12_	117.00	121.00	119.00	16.82	17.31	17.06	184.52	193.21	188.87	2.34 (1.69)	0.00 (0.71)	1.17 (1.20)
T_13_	120.00	124.00	122.00	17.02	17.74	17.38	188.03	196.97	192.50	2.60 (1.76)	0.00 (0.71)	1.30 (1.23)
T_14_	105.00	107.00	106.00	15.30	15.80	15.55	158.14	165.61	161.87	0.61 (1.05)	3.04 (1.73)	1.82 (1.39)
**SEm±**	**1.75**	**1.88**	**1.19**	**0.27**	**0.27**	**0.18**	**2.86**	**2.97**	**1.91**	**0.03**	**1.07**	**0.49**
**CD p = 0.05%**	**5.08**	**5.47**	**3.37**	**0.78**	**0.80**	**0.51**	**8.32**	**8.63**	**5.41**	**NS**	**NS**	**NS**

### Quality characteristics

The effect of organic manures upon fruit quality characteristics like juice percent (%) and total sugar (%) was recorded as significant, but fruit cracking percent (%) and rind thickness (mm) were found to be non-significant with organic manure application during investigation (Table 4 and Fig 5). The highest juice percent (52.33, 53.50 and 52.92%) and total sugar (11.86, 11.98 and 11.92%) were recorded with the organic combination T_13_-*Jeevamrut* 16.08 L plant^-1^ + Vermicompost 24.79 kg plant-1, which was on par with the treatment T_2_-RDF (600: 200: 200g NPK Plant^-1^ year^-1^) as compared to control T_1_ (nothing applied) during both the experimental years. For both juice percent and total sugars, overall significant trend in both years was as follows: T_2_> T_13_> T_12_> T_11_> T_9_> T_8_. For fruit cracking, overall most significant trend in both years was as follows: T_2_>T_13_> T_12_> T_11_> T_9_ > T_8_. For acidity, overall most significant trend in both years was as follows: T_2_>T_13_> T_12_> T_11_> T_8_ > T_5_.

**Fig 5:** The effect of different organic manure treatments on soil chemical properties, where (**a**) Juice percent; (**b**) Acidity percent; (**c**) Total sugars percent; d) Fruit cracking percent. Various asterisk on bars show the significant differences (*P* < 0.05) with vertical bars as standard errors (*n* = 4) (****>***>**>*>ns).

**Table 4:** Effect of organic manures on fruit quality characteristics of pomegranate cv. ‘Bhagwa’.

Treatment	Rind thickness (mm)			Juice percent (%)			Acidity (%)			Total sugar (%)		
	2019	2020	Pooled	2019	2020	Pooled	2019	2020	Pooled	2019	2020	Pooled
T_1_	3.48	3.74	3.61	48.66	49.20	48.93	0.51	0.51	0.51	10.80	10.99	10.89
T_2_	4.84	4.77	4.80	52.14	53.17	52.65	0.42	0.40	0.41	11.76	11.92	11.84
T_3_	3.73	3.84	3.78	50.33	51.00	50.66	0.46	0.45	0.45	11.06	11.16	11.11
T_4_	3.73	3.84	3.78	50.50	51.33	50.92	0.45	0.44	0.45	11.09	11.18	11.13
T_5_	4.00	4.04	4.02	51.00	51.90	51.45	0.44	0.44	0.44	11.17	11.27	11.22
T_6_	3.63	3.74	3.68	49.00	49.67	49.34	0.48	0.47	0.48	10.89	10.98	10.93
T_7_	3.63	3.74	3.69	49.33	50.10	49.72	0.47	0.47	0.47	10.99	11.08	11.03
T_8_	4.37	4.12	4.24	51.33	52.50	51.92	0.44	0.43	0.44	11.27	11.37	11.32
T_9_	4.70	4.59	4.65	51.50	52.67	52.09	0.43	0.42	0.43	11.43	11.54	11.48
T_10_	3.69	3.80	3.74	50.00	51.00	50.50	0.46	0.46	0.46	11.02	11.11	11.07
T_11_	4.47	4.20	4.34	51.67	52.90	52.29	0.42	0.42	0.42	11.60	11.72	11.66
T_12_	4.50	4.67	4.59	52.00	53.00	52.50	0.42	0.41	0.41	11.71	11.83	11.77
T_13_	4.77	4.72	4.74	52.33	53.50	52.92	0.41	0.39	0.40	11.86	11.98	11.92
T_14_	3.65	3.76	3.71	49.67	50.67	50.17	0.47	0.46	0.46	11.00	11.09	11.04
**SEm±**	**0.29**	**0.28**	**0.19**	**0.70**	**0.88**	**0.52**	**0.02**	**0.02**	**0.01**	**0.05**	**0.05**	**0.03**
**CD p = 0.05%**	**NS**	**NS**	**NS**	**2.04**	**2.55**	**1.48**	**NS**	**NS**	**NS**	**0.14**	**0.14**	**0.09**

## Discussion

The soil nutrient status at the termination of the experiment revealed that AN, AP, and AK content at different levels of organic amendments were affected significantly. The reason for this significant effect might be due to the fact that enhancement of basic soil properties is a long-term process. It is a well-known fact that incorporating organic manures into soils not only acts as a storehouse of major and micro nutrients, but also improves the soil’s physical, chemical, and biological qualities. These findings are consistent with those of Ghosh et al. (2010) [17] in pomegranate. Thus, organic manures’ potential role in crop growth can be attributed to its direct effect on the availability of essential plant nutrients, as well as the physico-chemical and biological properties of soils. In addition, organic manure also have indirect effect on the release of growth hormones, vitamins, and the expansion of microbial populations during its process of decomposition [5, 18]. Similar findings were reported in guava by Mitra *et al*. (2010) [19], and Devi *et al*. (2012) [20].

The increase in microbial count may be attributed to readily available micronutrients and organic manures as sources of organic carbon for microbial population buildup. It may also be attributed to favourable excretions by root exudates like carbohydrates, amino acids, organic acids, and many growth promoting substances that act as food substrates for microbes [21]. Unlike FYM, vermicompost establishes a suitable environment for microbes and worms to flourish. During vermicomposting, earthworms ingest plant growth promoting rhizosphere (PGPR) bacteria such as *Rhizobium*, *Bacillus*, etc. along with rhizospheric soil, and they might get activated or increased due to the ideal microenvironment of the gut. Therefore, the population of PGPR gets a boost from the earthworm’s activity [22]. The elevated amounts of microbial biomass in the soil may be due to increased levels of implementation of various organic manures, which provide appropriate biomass as a feed for microbes and aid in the expansion of the microbial population in the soil [23]. In addition, vermicompost has a large specific surface area, which provides a large number of microhabitats for microbial activity.

For most soil organisms, organic matter is the primary source of energy and food. It has a huge impact on the general microbial population. Differential microbial population stimulation is caused by the type of organic material. Organic matter affects the structure and texture of soil, as well as providing nutrients to plants and microorganisms. The activity of soil microorganisms is also influenced by such factors in the soil. H-ion concentration is a key factor influencing the microflora of soil. This greatly influences the enzyme system and thus plays an important role in microbial activity [24]. There are several direct and indirect effects of H-ion and salt concentration in soil on the microbial population [25]. Thus, every direct and indirect change in crop production may result in altering the soil microflora. But all these changes seem to be only temporary, as very often the microbial equilibrium is restored to the original level.

The result shows that the inorganic fertilizer significantly promoted the yield characteristics, which was statistically on par with organic manures. The improved outcomes of inorganic fertilizer were attributable to a greater supply of important plant nutrients, which are needed in greater quantities for plant growth and development. The optimal administration of nitrogen resulted in the faster development of the growth and reproductive phases. Furthermore, greater nitrogen levels may have expedited protein synthesis, allowing for earlier floral primordial development. As a result, an increase in phosphorus is implicated in the onset of floral primordial development, resulting in an increase in the number of flowers and fruits per plant. In previous studies, it was found that the yield of pomegranate plants was significantly increased with different levels of nitrogen [26]. Vermicompost outperformed the other organics in terms of growth, which could be due to the readily available and increased nutrient content in vermicompost. The improved growth could also be attributed to improved moisture retention and nutrient availability as a result of the favourable soil conditions created by vermicompost treatment. Improved nutrient uptake, carbohydrate synthesis, translocation, and hydration status of plants may have helped the plants put up greater vegetative growth and flowering, as well as a high fruit set, resulting in a greater number of fruits per plant and yield. Organic manure nutrients were released slowly and made available throughout the growth period, resulting in improved nutrient uptake, plant vigour, and yield. Enhancement of the microbial population and improved soil physical environment may have made it easier to absorb nutrients in a balanced form, resulting in higher production. In previous studies, it was found that application of poultry manure recorded the highest fruit yield in pomegranate [27]. Similar results were observed in Assam lemon [28].

The availability of nutrients may have boosted photosynthate production, translocation, and accumulation in the sink. This may have prompted the plants to produce more fruitful buds, resulting in a greater okra fruit yield and more fruits per plant. It was also recorded that the increase in the number of fruits owing to this treatment might be due to the greater availability of mineral nutrients from the nitration of vermicompost [29]. Jeevamrut’s favourable benefits were linked to a larger microbial load and growth hormones, which may have increased soil biomass, hence maintaining the accessibility and absorption of applied and native soil nutrients, resulting in improved capsicum growth and production [9, 30]. The liquid manures (*Panchgavya*, *Jeevamrut*, and *Sanjeevak*) provide balanced nutrition to the crops and help to improve the yield as they provide readily available nutrients, growth hormones, and microbes to *Vigna radiata*. In one of the studies, it was concluded that *Jeevamrut* contains an enormous amount of microbial load which multiplies and acts as a soil tonic [31]. Its use boosts microbial activity in the soil, ensuring nutrient availability and uptake by crops. It boosts soil biological activity and increases crop nutrient availability, and it is a low-cost impromptu preparation that helps mineralization by enriching the soil with indigenous microorganisms. Greater output on a number and weight level might be ascribed to improved amounts of nutrients in the crop’s absorbing region, which increased production. Similarly, the yield qualities enhanced as a result of sensible partitioning of the economic sink [32]. Increased fruit weight and productivity due to organic manure treatment may be responsible for plant growth hormone synthesis, root system development, and hence high nutrient use by crop plants in cape gooseberry [33] and tomato [34].

In comparison to inorganic fertilizer, the application of organic manures had a considerable impact on the quality features of pomegranates. Because organic manures, such as vermicompost, contain important nutrients in conveniently accessible forms, they promote plant growth by giving vital nutrients to plant physiological activities. The application of vermicompost improved the soil’s physico-chemical characteristics, enzymatic activity, and microbial population. The increase in fruit quality could be attributed to a better supply of micronutrients and hormone stimulation, which improves cell division and elongation, fruit size and weight, root growth, water uptake, and nutrient deposition. Increased N addition and catalytic activity of numerous enzymes could possibly be the reason [28]. Organic sources were used to increase the quality characteristics. This could be attributed to improvements in soil physical and biological properties. Increased soil conditions may have improved pomegranate root growth, nutrient uptake, and quality. Application of nutrients in the form of vermicompost and Jeevamrut mixture improved the qualitative attributes of organic sources.

In general, the quality of the fruit juice produced with organic manure was superior to that generated with inorganic fertilizer. Under south Indian circumstances, elevated leaf K levels resulted in improved pomegranate fruit quality [27]. Increases in tomato quality metrics could be attributed to increased accessibility of major and minor nutrients, particularly nitrogen and potassium, which are important in improving fruit quality, while decreases could be owing to a lack of essential nutrients [35]. Potassium’s effect on fruit quality can be explained by the fact that it increased photosynthetic activity and aided in metabolite transfer from leaves to fruit [36].

The addition of organic manures provides adequate nutrients, moisture, and growth-promoting compounds, which boosts the plant’s metabolic and hormonal activity and encourages the creation of additional photosynthates, which are stored in the fruits as starch and carbohydrates. It is a well-known observation that the transition of mature fruit into ripe form, i.e., the fruit experiences physical, physiological, and biochemical changes. The conversion of conserved starch and other insoluble carbohydrates into soluble sugars could explain the increase in the total sugar content of papaya fruits. The positive influence of boron and zinc in the conversion of acids into sugar and their derivatives by the reaction involving the glycolytic pathway or being used in respiration in both fruit crops may be due to the positive influence of boron and zinc in the conversion of acids into sugar and their derivatives by the reaction involving the glycolytic pathway or being used in respiration in both fruit crops [37]. Previous research in guava suggests that increased fruit quality characteristics are attributable to the addition of various organic manures and amendments to the soil and, as a result, to the plants, which may have promoted the biosynthesis and translocation of carbohydrates into the fruits [38]. Furthermore, because of the increased rate of photosynthesis, the accessibility of nitrogen from various sources may have enhanced the leaf area with higher assimilate synthesis. Such effects have been related to an increase in the rate of photosynthetic product translocation from leaves to developing fruits, resulting in a rise in total sugars. Similar results have also been reported by Singh *et al*. (2015) [39] in strawberry.

## Conclusion

The conclusion of this experiment is that the use of organic sources has been more helpful in increasing the nutritional as well as microbial status of the soil. The combination of Jeevamrut (16.08 L/plant) and Vermicompost (24.79 kg/plant) improves the nutritional status as well as the microbial population of the soil in the pomegranate cv. Bhagwa field. It may also be concluded that the application T_13_-*Jeevamrut* 16.08 L plant^-1^ + Vermicompost 24.79 kg plant^-1^ enhanced fruit yield characteristics like fruit plant^-1^ (122.00), fruit yield (17.38 kg plant^-1^), fruit weight (192.50 g), and fruit quality characteristics such as fruit juice percent (52.92%), and total sugar (11.92%). Based on the findings, pomegranate growers could be advised to use an organic combination of Jeevamrut 16.08 L plant^-1^ + Vermicompost 24.79 kg plant^-1^ to improve the yield and quality characteristics of pomegranate fruits, as well as to improve the nutritional status and microbial population of the soil, which aids in the growth, yield, and quality of pomegranates.
